# Arthroscopic partial trapeziectomy and tendon interposition for thumb carpometacarpal arthritis

**DOI:** 10.1186/s13018-015-0329-y

**Published:** 2015-12-18

**Authors:** Min-Yao Chuang, Chang-Hung Huang, Yung-Chang Lu, Jui-Tien Shih

**Affiliations:** Department of Orthopaedic Surgery, MacKay Memorial Hospital, No. 92 Sec. 2 Zhongshan N. Rd., Taipei City, Taiwan; Department of Medical Research, MacKay Memorial Hospital, New Taipei City, Taiwan; Department of Dentistry, National Yang-Ming University, No. 155 Sec. 2 Linong St, Taipei City, Taiwan; Department of Cosmetic Application and Management, MacKay Junior College of Medicine, Nursing, and Management, No. 92 Shengjing Rd, Taipei City, Taiwan; Department of Orthopaedic Surgery, Taoyuan Armed Forces General Hospital, No. 168 Zhongxing Rd, Longtan District Taoyuan City, Taiwan

**Keywords:** Thumb carpometacarpal joint, Arthroscopic, Arthritis, Trapeziectomy, Level of evidence: level IV

## Abstract

**Background:**

The purpose of this study was to introduce arthroscopic partial trapeziectomy and tendon interposition for the treatment of symptomatic thumb carpometacarpal arthritis of Eaton stage II or III.

**Methods:**

From August 2001 to April 2009, 23 patients with thumb carpometacarpal arthritis were treated using this technique. Pain score, range of motion, and pinch strength were clinically evaluated and compared with the preoperative values after a minimum follow-up duration of 24 months.

**Results:**

Significant reduction in pain score and increases in range of motion and pinch strength were found (all *p* < 0.001) after a 2-year follow-up. The mean ± SD (median) postoperative pain score was 1.0 ± 0.7 (1.0) at rest and 1.3 ± 0.9 (1.0) during daily activities. The postoperative range of motion was 19.1° ± 4.2° (20°) for extension and 35.7° ± 7.1° (35.0°) for flexion, and the postoperative pinch strength was 86.5 % ± 19.9 % (90.0 %). No complications were observed in our patient series.

**Conclusions:**

Arthroscopic partial trapeziectomy and soft tissue interposition could be an alternative treatment method for patients with symptomatic thumb carpometacarpal arthritis of Eaton stage II or III.

## Background

Thumb carpometacarpal (CMC) joint arthritis is a common disease and usually affects women in the postmenopausal age group [1–3]. Typical conservative treatment includes functional education, activity modification, anti-inflammatory medications, intra-articular steroid injections, and splinting. The indication for operative intervention is failure of conservative treatment. Numerous surgical techniques have been described, including ligament reconstruction and tendon interposition (LRTI) [4], suspensionplasty [5], first metacarpal extension osteotomy [6], arthrodesis [7], hematoma distraction arthroplasty [8], artificial prosthesis replacement [9], osteochondral allografting [10], hemitrapeziectomy [11], complete trapeziectomy [12], arthroscopy [13], volar ligament reconstruction [14], and various combinations of these procedures. The most common surgical treatment currently used is trapezium excision combined with LRTI [4].

The specific types of surgical procedures for thumb CMC joint arthritis are usually divided between those for Eaton stage I and II–IV disease, depending on whether the cartilage of the basal joint remains unaffected or has existing evidence of degeneration [15].

Procedures for stage I disease include volar ligament reconstruction, arthroscopy, and first metacarpal extension osteotomy. Volar ligament reconstruction has the advantages of halting the radiographic progression of the disease and the disadvantage of relatively poor pain relief. Arthroscopy is a less invasive procedure and can be used simultaneously in the treatment of ligament laxity. First, metacarpal extension osteotomy has the benefit of correction of an adduction contracture but is associated with the possibility of nonunion and implant problems.

For stage II–IV disease, surgical treatment options have evolved over the past 50 years, including trapeziectomy, hemitrapeziectomy, arthrodesis, artificial prosthesis replacement, LRTI, suspensionplasty, osteochondral allografting, and hematoma distraction arthroplasty. Simple trapeziectomy/hemitrapeziectomy has the advantages of decreased operative time, pain relief, and minimal donor site morbidity. Its disadvantages include significant functional problem and loss of pinch strength. Arthrodesis is mainly performed in workers with heavy workload and cases of posttraumatic arthritis in young patients and as a salvage procedure for failed reconstructive surgery. Although this technique preserves pinch strength, concurrent problems occur, including nonunion, degenerative changes in neighboring joints, and loss of mobility. The artificial prosthesis replacement procedure shows good short-term results [9], but its application is diminished by reports of prosthetic failure, instability, foreign body synovitis, cold flow, and wear debris. With high patient satisfaction and preservation of function, LRTI has increased in popularity and is considered by many to be the standard surgical procedure for these cases. Suspensionplasty is an easier procedure with several advantages, including decreased deforming force of the abductor pollicis longus, preservation of the flexor carpi radialis, and release of both the first dorsal compartment and the more distal position of the suspension. Disadvantages include possible injury to the superficial radial nerve and a cosmetically unappealing bump. Osteochondral allografting has shown promising short-term results, but with problems of allograft fracture and infection. Hematoma distraction arthroplasty is a less complicated procedure but with similar good results. However, metacarpal subsidence is a frequent concern.

We introduced arthroscopic treatment of stage II and III disease to achieve a minimally invasive surgery [13]. In addition, partial trapezium resection and interposition arthroplasty have been used to preserve stability [11]. It is hypothesized that partial resection of the trapezium combined with thermal shrinkage of the volar ligaments and capsule, soft tissue interposition with palmar longus tendon, and temporary K-wire fixation for support, performed with the aid of arthroscopy, would be an alternative technique for the treatment of stage II and III thumb CMC joint arthritis.

## Methods

### Patient cohort

Our institutional review board approved this study. The study included all patients treated between August 2001 and April 2009 whose conditions required surgical intervention and who met the inclusion criteria. Patients with symptomatic Eaton stage II or III thumb CMC joint arthritis based on preoperative radiographs (Fig. 1a) and previous failure of at least 6 months (range, 6–12 months) of conservative treatment were included in this study. Conservative treatment included a regimen of rest, thumb brace, activity modification, nonsteroidal anti-inflammatory medications, and a mean of two cortisone injections (range, one to six injections). Patients with previous thumb trauma and other concomitant diagnoses that probably caused confusion in the diagnosis and affected the interpretation of the results (e.g., Bennett’s fracture and de Quervain’s tenosynovitis) were excluded. As a result, 23 patients (23 thumbs) were included in this study. The patients underwent arthroscopic partial trapeziectomy and interposition of the palmar longus tendon. Of the 23 patients, 3 were men and 20 were women, with a mean age of 59.0 years (range, 54–68 years), and 10 had Eaton stage II disease and 13 had stage III disease. All the patients were right-hand dominant, and only two patients underwent surgery for nondominant thumbs. The medical conditions of the old patient group were allowed surgical treatment.

**Fig. 1:** **a** Preoperative radiographic images demonstrating Eaton stage III osteoarthritis of the right thumb carpometacarpal joint. **b** Immediate postoperative radiograph showing a K-wire used for fixation across the thumb carpometacarpal joint. **c** Radiographs obtained at 24 months after surgery showing a stable thumb carpometacarpal joint

### Surgical technique

All of the operations were performed under general anesthesia and tourniquet control. A single finger trap was used on the thumb with 5 to 10 lb of longitudinal traction by using a traction tower. The CMC joint was identified and localized by palpation or fluoroscopy. Two incision portals were marked. One was located radial to the first extensor compartment tendons, while the other was ulnar to the first extensor compartment tendons along the line of the joint. The distance between each portal and insertion of the first extensor compartment tendons was about 1 cm (Fig. 2). The radial portal was used for assessment of the joint cartilage, as well as the dorsoradial, posterior oblique, and ulnar collateral ligaments. The ulnar portal was helpful for treating and visualizing the volar ligaments. Joint distension with 2 to 3 mL of normal saline solution facilitated the placement of a 1.9-mm, 30° short-barreled arthroscope. A full-radius mechanical shaver and a burr with suction were used for debridement and partial trapeziectomy (Fig. 3a). Ligamentous laxity and capsular attenuation were treated with thermal capsulorrhaphy with a radiofrequency shrinkage probe (Fig. 3b). The Oratec MicroTAC-S probe (MicroTAC-S, Oratec Interventions, CA) was inserted through the portals and used at a setting of 67° and 40-W power. The probe was gently swept over the volar ligaments. Radiofrequency energy was applied slowly and deliberately to allow tissue shortening and blanching to be visualized. A 10-cm-long tendon graft taken from the palmar longus tendon (Fig. 4a) was rolled and sutured into a ball measuring approximately 1 cm in diameter (Fig. 4b). The ball was pushed into the CMC joint via the portal (Fig. 4c). The correct position of the ball was confirmed under arthroscopy, and the tendon ball was subsequently anchored to the capsule by absorbable sutures. A 1.2-mm K-wire was used for fixation across the CMC joint (Fig. 1b), and a short-arm thumb spica splint was applied. The sutures were removed after approximately 10 postoperative days, and a short-arm cast was applied for an additional 4 weeks, at which time the pin was removed. Formal occupational therapy was started, and a removable brace was worn for an additional 4 weeks.

**Fig. 2:** Intraoperative image demonstrating the *radial* and *ulnar portals* of arthroscopy

**Fig. 3:** Intraoperative arthroscopic images. **a** Arthroscopic view of a 2.0-mm burr that was used to partially remove the trapezium. **b** Arthroscopic view demonstrating thermal shrinkage of the volar ligaments (AOLs) with the use of a radiofrequency electrothermal probe

**Fig. 4:** **a** The palmar longus tendon is harvested by a tendon stripper. **b** The tendon graft is rolled into a ball. **c** The tendon ball is pushed into the basal joint using the portal

### Clinical evaluations

#### Preoperative assessment

All patients complained of preoperative pain at the thumb base that impaired performance of daily activities. Physical examinations of the patients included an assessment of the thumb CMC joint range of motion (flexion and extension) with a protractor goniometer (Fig. 5b), determination of the site of tenderness and pain by using a 10-point visual analog scale (VAS), axial stress grind test, and the identification of the thumb pinch strength with a Jamar dynamometer (Therapeutic Equipment, Clifton, NJ, USA). Plain radiographs of the thumbs were obtained from all patients (Fig. 1a).

**Fig. 5:** **a** Schematic diagram showing the range of motion of the thumb carpometacarpal joint at postoperative follow-up. **b** Measurement of range of motion

#### Postoperative assessment

Each patient was assessed clinically at 2, 3, 6, 12, and 24 months after surgery. After 24 months, they returned for evaluation according to their own volition. The assessment included pain (VAS score), thumb pinch strength measured with a Jamar dynamometer, and thumb CMC joint range of motion (Fig. 5a). The presence of any complications was also recorded. Standard anteroposterior and lateral radiographs of the thumb were also obtained during each assessment and used to ensure that the CMC joint had not subluxated or collapsed (Fig. 1c).

#### Statistical analysis

Statistical analysis was performed with the SPSS software (SPSS version 10.0, Chicago, IL, USA). Continuous data were presented as mean ± SD. Categorical variables were presented as frequency (%). The Wilcoxon signed-rank test was used to compare postoperative thumb pain, range of motion of the thumb CMC joint, and thumb pinch strength with the preoperative measurements. Statistical significance was defined as a *p* value <0.05.

## Results

At enrollment, the mean pain scores at rest and during daily activities were 5.7 ± 0.5 (median, 6) and 7.0 ± 0.6 (7.0), while the extension and flexion ranges of motion (ROMs) and pinch strength were 15.9° ± 3.9° (15.0°); 27.8° ± 8.2° (30.0°); and 47.2 % ± 9.4 % (50.0 %), respectively. The data of the clinical outcomes are summarized in Table 1. None of the patients required or opted for further surgery of the thumb, and improvements in all parameters (i.e., pain score, ROM, and pinch strength) were observed after the operations. Significant reduction in pain score and increases in the ROM and pinch strength were subsequently observed (all *p* < 0.001). The mean postoperative pain score was 1.0 ± 0.7 (median, 1.0) at rest and 1.3 ± 0.9 (1.0) during daily activities. The postoperative ROM was 19.1° ± 4.2° (20°) for extension and 35.7° ± 7.1° (35.0°) for flexion, and the postoperative pinch strength was 86.5 % ± 19.9 % (90.0 %).

**Table 1:** Preoperative and postoperative outcomes of the patients

Outcomes	Preoperative (*n* = 23)	Postoperative (*n* = 23)	*p* value
Pain at rest (points)	5.7 ± 0.5	1.0 ± 0.7	**<0.001**
			**(1.948E-5)**
Pain during daily activities (points)	7.0 ± 0.6	1.3 ± 0.9	**<0.001**
			**(2.330E-5)**
Extension ROM (degrees)	15.9 ± 3.9	19.1 ± 4.2	**<0.001**
			**(2.750E-4)**
Flexion ROM (degrees)	27.8 ± 8.2	35.7 ± 7.1	**<0.001**
			**(1.58E-4)**
Pinch strength (%)	47.2 ± 9.4	86.5 ± 19.9	**<0.001**
			**(2.548E-5)**
Proximal subsidence of the metacarpal shaft (mm)	**-**	2.1 ± 0.9	**-**

*Abbreviations*: *ROM* range of motion

Data were presented as mean ± SD and analyzed using the signed-rank test. Values with bold emphasis indicate a significant change after surgery (*p* < 0.05). The dash denotes the same data and that no comparisons were needed

None of the patients who underwent the procedure had infections or other complications. All patients were satisfied with the surgical results within three postoperative months. Follow-up radiographs obtained at 24 postoperative months were compared with the immediate postoperative radiographs and demonstrated a mean proximal subsidence of 2.1 mm (0–4 mm) of the metacarpal shaft (Table 1). No cases of radiographic basal joint subluxation or scaphotrapezium joint arthritis were found.

## Discussion

Small joint arthroscopy for the smaller joints of the hand, first introduced by Watanabe [16], has been refined over the years by other authors [17, 18]. Arthroscopy of arthritic thumb CMC joint, a minimally invasive procedure first described by Menon [19], allows for joint visualization, treatment, and disease staging. Furia [20] described his experience with arthroscopic debridement and synovectomy in a series of 23 patients with stage I and II disease. Good or excellent results in terms of pain relief, functional scores, subjective outcomes, and pinch strength were reported in 83 % of the surgical patients. Arthroscopy is currently considered reliable for the evaluation and treatment of thumb CMC joint arthritis [13]. Our study introduced arthroscopic treatment for patients with Eaton stage II or III thumb CMC arthritis.

The stability of the thumb CMC joint depends on static ligamentous restraints because of the lack of bony congruity [21]. Laxity of the ligaments has been proposed as a mechanism of the development of thumb CMC joint osteoarthritis [22]. Thus, addressing joint instability is a vital component of surgical treatment. The anterior oblique ligament is believed to be the primary stabilizer. This belief is supported by the clinical success of the reconstructive procedures for this ligament [23]. In order to recreate this ligament, researchers have used several methods, which are technically challenging. Electrothermal shrinkage would be an alternative simple method for the treatment of volar ligament laxity [24]. In this study, we selected this surgical technique to minimize damage of soft tissues.

Total excision of the trapezium results in good pain relief but also in substantial loss of thumb strength and stability [25]. To avoid the negative results, many surgeons have elected to excise just the articular surface of the trapezium [26, 27]. In our patients, hemitrapeziectomy was conducted to avoid these sequelae.

After hemitrapeziectomy, interposition arthroplasty preserves the stability of the thumb CMC joint by maintaining the joint space [4]. The best interpositional material is an autologous tendon graft, and it is important to pack the joint space with as much tendon as possible to keep the first metacarpal and trapezium apart. The tendon ball should be larger than the removed bone. In addition, bleeding from the subchondral bone fills the interspaces of the coiled tendon graft. The clot then organizes and is eventually converted into fibrous tissue that acts as a spacer, keeping the opposing bones apart. In the present study, interposition arthroplasty with a palmar longus tendon graft was chosen to help improve stability.

Long-term clinical studies on arthroscopic hemitrapeziectomy with interposition arthroplasty have not been well reported in the literature. Pegoli et al. [28] evaluated the clinical outcomes of 16 patients with Eaton stage I and II arthritis and reported that 12 of these patients had good to excellent results at a mean follow-up period of 12 months. In addition, Earp et al. [29] investigated a similar procedure in patients with stage II and III arthritis and a mean follow-up period of 11 months. They observed improved pain scores and a high rate of patient satisfaction. In our series of 23 patients, pain score, pinch strength, and range of motion significantly improved after a minimal postoperative period of 24 months, which was longer than those in previous studies.

Furthermore, in our previous study [24], we recorded pain scores, range of motion, and pinch strength of the thumb to assess clinical outcomes of arthroscopic thermal treatment in patients with Eaton stage I and II arthritis. Significant improvement was observed in pain score during daily activities, in flexion ROM, and in pinch strength after surgery at a mean follow-up period of 24 months. In the present study, we further modified the surgical procedure to treat patients with stage II and III arthritis by using the same evaluation methods. Hemitrapeziectomy and tendon interposition were added to the treatment procedures for the patient group with advanced disease stage. Although the clinical evaluation methods used in each study varied, these simplified evaluation methods might provide relatively objective information to demonstrate the possibility of using this surgical procedure for the treatment of patients with Eaton stage II or III symptomatic thumb CMC arthritis.

The present surgical method is less invasive than the conventional open method. The capsule is not destroyed during the procedure, and a closed space is maintained for true soft tissue interpositional arthroplasty. Furthermore, this reduces the chance of damage to the radial sensory nerve branch. However, this procedure is technically demanding and could require longer operation time. This approach may not be suitable for patients with mild stage I and severe stage IV disease. Hemitrapeziectomy is unnecessary, and arthroscopic treatment alone is enough for patients with stage I disease. It could be contraindicated for patients with stage IV disease. An open procedure would be beneficial for patients with severe disease.

This study has some inherent limitations. First, the number of patients was small, and the male to female patient ratio in the group was less than that reported previously [1–3]. Second, the study was a retrospective review with intermediate follow-up. Moreover, we did not administer a questionnaire to assess function and conduct a test to assess grip strength, range of motion with abduction/adduction, and which crease the thumb can reach.

## Conclusions

Arthroscopic partial trapeziectomy and soft tissue interposition could be an alternative treatment method for patients with Eaton stage II and III symptomatic thumb CMC arthritis. Longer-term follow-up would be more helpful to validate the superiority of this procedure to the conventional approach.

## Abbreviations

CMC: carpometacarpal
SD: standard deviation
VAS: visual analog scale
